# Neural Network Model for Perceptual Evaluation of Product Modelling Design Based on Multimodal Image Recognition

This article has been retracted.

**DOI:** 10.1155/2022/1665021

**Published:** 2022-08-09

**Authors:** Jie Wu, Long Jia

**Affiliations:** ^1^School of Anyang Institute of Technology, Anyang, Henan 455000, China; ^2^Anyang Institute of Technology, School of Art and Design, Anyang, Henan 455000, China

## Abstract

With the homogenization of product function and performance, the design technology for product appearance quality has been increasingly valued by academia and industry and has become an effective technical way to meet the continuously growing diversified and personalized needs of consumers. The appearance quality attribute of a product can be characterized or described by its appearance image. Data-driven product appearance image design is based on the quantitative data of product appearance and consumer emotional needs and completes the product appearance through computer-aided design technology and intelligent algorithms. Design innovation can help companies quickly respond to consumers' emotional needs and effectively improve design quality and product competitiveness. When visual objects are disturbed in complex scenes, the issues such as how the human brain coordinates multisensory information processing and what neural processing mechanisms follow are still unclear. In this paper, a visual object recognition experiment in a complex scene was designed and the brain activation signals of three modalities of noise, added audio-visual (AVd), single visual noise and noise (Vd), and single-audio (A), were recorded. The properties and neural processing mechanisms of multisensory modulation of auditory stimuli during noisy image recognition were explored. Using the conjunction method combined with the classic “max criterion” rule, it was found that only when a certain amount of noise was added to the visual stimulus, the integration area changed. The product appearance has a decisive influence on the user's product perceptual attribute preference and greatly affects the consumer's satisfaction. The importance of product appearance image design is increasingly prominent. In addition, pattern analysis of brain activation signals confirmed that semantically consistent sounds can facilitate the recognition of noisy images and this facilitation shows a certain category selectivity when subdivided into categories. Using the analysis method of functional connectivity, a functional connectivity network containing nodes at different integration levels was constructed to explore the overall characteristics and processing patterns of the multisensory network. Through the analysis of the network connection relationship, it is found that the prefrontal cortex, STS, and lateral occipital lobe are the nodes with more aggregation in the network, and their functions are similar to the hub in the network. The brain functional network was constructed, and functional connectivity was used to explore the connection characteristics of the network and the multisensory modulation mechanism between different processing levels of the brain.

## 1. Introduction

With the advancement of science and technology, the development of economy and culture, and the improvement of consumers' living standards, the market competition has become increasingly fierce and product quality has become the key to winning the competition of enterprises. The quality of a product is characterized or described by its specific quality attributes. Modern products usually contain two quality attributes, namely, the objective attributes embodied in the function and performance of the product and the perceptual attributes conveyed by the shape and color of the product. The literature believes that modern products must have richer emotional expression, and the perceptual attribute has become an important attribute of modern industrial products. Consumers' demands for products are becoming more and more complex and diverse, and among many demands, functional and perceptual demands are crucial to improving consumer satisfaction [1]. The quality attributes of products are given by specific design technologies and through specific design processes. Due to the increasing maturity and convergence of product technologies, there is a lack of effective technical barriers among competitors and it is difficult to appear in a fully competitive market based on function. The competitive advantage formed by design is that the formation of product attractiveness is no longer simply to provide functions, but to effectively express the perceptual attributes of products [2]. Therefore, expressing the perceptual attributes of products accurately, timely, and effectively through design has become an indispensable and important way to improve the quality attributes of products and consumer satisfaction. Product image is a concentrated reflection of people's psychological emotions and product perceptual attributes formed by a product and contains rich product perceptual information. So far, it has become an important medium to improve product design quality and consumer satisfaction [3].

The product appearance has a decisive influence on the user's product perceptual attribute preference [4] and greatly affects the consumer's satisfaction. The importance of product appearance image design is increasingly prominent [5–7]. It aims to effectively convey the perceptual attributes of products and endow products with higher perceptual quality and plays an important and positive role in the development of products that integrate innovation and satisfaction. At present, the key technical theory used to build the bridge between product appearance and product image is the theory of Kansei Engineering, which has achieved considerable success in the field of industrial design [8]. As the main design research theory for product appearance innovation, Kansei Engineering combines specialized knowledge in statistics, mathematics, and computer fields to acquire and process consumers' emotional needs, so as to establish objective data relationship and relationship between product appearance and its imagery. It is possible to form data-driven quantitative research on product appearance image design and help designers complete product appearance image design more scientifically and efficiently [9]. The essence of “image” is a kind of conscious activity in which objective things are perceived by people's perception system and associated with information transmission, which condenses people's inner feelings and emotional responses to the characteristics and attributes of things [10]. After being triggered by an object, the human perceptual system will form a certain perceptual image of the object and express it through perceptual image adjectives such as “modern, dynamic.” Image triggers include visual, tactile, and auditory pathways, among which vision is the most important way to form and convey images, and it also constitutes the main theoretical basis for image design with product appearance as the core [11]. Product appearance is mainly composed of shape and color, which are two key visual elements that determine the image of product appearance [12]. Shape and color work together on the user's visual perception system and trigger an emotional response, which makes it form an overall perceptual image of the product's appearance and generate purchase behavior. Therefore, the image design of shape and color represents the two core contents of product appearance image design and is applied to a wide range of product fields.

In this paper, we want to explore the multisensory modulation effect of semantically consistent sounds on image recognition in the case of visual image noise. Therefore, the experiment should include the conditions of three modalities (mono-audio, mono-vision, and audio-visual integration) and also consider category conditions in cognitive tasks. This paper adopts the factor block experiment paradigm, which not only meets the requirements of cognitive tasks but also provides a basis for data processing in different ways. This paper uses multimodal image recognition technology to study the multisensory modulation mechanism of auditory stimuli in noise image recognition, trying to explore the processing characteristics of different integration areas in the process of multisensory modulation and the relationship between them. Cognitive laws and neural mechanisms are exhibited at different processing levels. First, this paper designs a task-state factor chunking experimental paradigm, considering three modalities of audio-visual, audio-visual, and audio-visual integration simultaneously to explore the modulation effect of auditory information on visually noised images. Second, the classical “max rule” combined with univariate analysis was used to investigate the changes and performance characteristics of key integration regions and the method based on multivoxel pattern analysis was used to decode visual objects at different class levels. Next, by constructing a brain network of key integration nodes, we examine the interaction and regulatory mechanisms between these integration regions. Finally, in order to comprehensively investigate the multimodal information processing mechanism, the integration nodes were located in multiple processing levels, the brain functional network was constructed, and functional connectivity was used to explore the connection characteristics of the network and the multisensory modulation mechanism between different processing levels of the brain.

## 2. Related Work

At the beginning of the last century, researchers began to study the behavioral characteristics of multisensory information integration and processing. It is typical to combine visual and auditory information to test the response time of the subjects to stimuli, and it is found that the response time of the subjects is significantly lower than that of a single stimulus combination of multimodal stimuli [13]. By combining the changes of the visual ring with the changes of the auditory stimuli in pure tone decibels, a selective property in the integration of multisensory information was found, that is, the closer the combination of visual and auditory stimuli, the faster the response time of the subjects. Similar experimental conclusions were also obtained in the experiments of multisensory information integration in animals. For example, using mice as research subjects and presenting them with various combinations of visual and auditory stimuli, the results showed that the reaction time of the mice to consistent visual and auditory stimuli was shorter than that of other single-modal stimuli. In addition, this conclusion has also been confirmed in studies of advanced primates. The researchers presented monkeys with visual (flash) and auditory (noise) stimuli and found that the behavioral response of the monkeys to the combination of flash and noise was significantly faster than a single stimulus. The above studies all show that whether in animals or humans, multisensory information processing shows the response advantage of multimodal processing in behavior, that is, compared with modalities, multimodal information integration has higher response time and accuracy rate. Many important findings at the neuronal level for the integration of multisensory information have been found in animal models. The superior colliculus is the first brain integration area to be studied in animal models. This area is considered to be the first area where multisensory information channels converge. Damage to this area will lead to the loss of multisensory information and the decline of integration function. In addition, this area is also a behavioral area, the region where the reaction starts [14–16].

A classic multimodal experiment was designed, allowing cats to receive visual, auditory, and tactile stimulation information, respectively, and to record the neuron firing activity in the superior colliculus. They found that when the cat received multisensory stimulation, the neurons in the superior colliculus fired. The ratio is significantly higher than the sum of the linear superposition of neuron firing ratios in a single modality. Subsequently, the neuron firing activity of the integration of multisensory information on the superior colliculus was subdivided, and it was found that the neuronal activity of the superior colliculus contains two multisensory information processing modes of enhancement and inhibition, and one may appear in the case of weak stimulation. The phenomenon of strong neuron firing activity is called the reversal effect [17]. Quantitative mathematical description based on product appearance requires comprehensive and accurate reflection of appearance characteristics, which is the basis and precondition for data-driven product appearance image design research. The mathematical model of product appearance quantification is the key to ensure the quality of appearance data. The currently used mathematical models have shortcomings such as the accuracy, comprehensiveness, and applicability of image-oriented appearance quantification, lack the ability to refine and complete the description of appearance feature information, and ignore the data fusion between different data and the relationship between different design links [18–20].

Product two-dimensional modeling is an important research object in the field of product image modeling design. From the perspective of product modeling description, the 2D modeling line has the advantages of adequacy of modeling description relative to points and operability relative to modeling description of surfaces [21]. Among them, the key modeling feature line can better characterize the important features and main styles of product modeling. Therefore, the quantitative mathematical description of product two-dimensional modeling is generally carried out with the key modeling feature line as the object. The commonly used two-dimensional modeling quantitative technology methods mainly include the curve control method, morphological analysis method, and harmonic analysis method [22]. Among them, the curve control method and the morphological analysis method have the deficiencies explained above. The mathematical model of the product 2D modeling quantification constructed in this paper is mainly realized based on the elliptic Fourier technology in the harmonic analysis method. The model construction process is as follows: first, digital image preprocessing is performed on the product modeling image, the boundary coordinates of the modeling contour are extracted, and the coordinates are converted into complex coordinate functions; then, a standardized new interpolation point coordinate sequence is generated by equidistant interpolation. The leaf series expands the sequence, calculates the ellipse Fourier coefficient matrix that can describe and reconstruct the shape contour, and finally obtains the principal component data through the principal component analysis of the matrix and completes the refinement of the shape contour information.

## 3. Multimodal Image Recognition

### 3.1. Multimodal Integration Activation Area

In the behavioral results, the semantically consistent sounds can help the subjects to accurately recognize the noised pictures, which shows that the semantically consistent sounds have a facilitation effect on the recognition of the noised pictures. To further verify whether the activation pattern of brain activity also has this facilitation effect, we examined the differences in the classification accuracy and dissimilarity values of AVd modal and Vd modal according to the hierarchical classification. In the coarse class grouping, both the RDM and classification accuracy of the AVd modality are significantly higher than those of the Vd modality (see Figure 1). These results further validate the facilitation of semantically consistent auditory stimuli in the recognition of noisy images. In order to exclude the influence of the number of voxels on the verification facilitation in the multivoxel pattern classification method, that is, the number of voxels in the selected brain regions may have an impact on the classification results of different modalities, we select the top 30, 60, 90, 120, 150, 180, and 210 voxels with the highest cumulative contribution rate, respectively, for the BA18 and STS/STG regions under the coarse and fine groupings as features for classification. Under the fine grouping, the classification accuracy of the BA18 region was significantly higher than that of the STS/STG region in both AVd and Vd modalities. In a similar recent cross-modal fMRI study, researchers were able to infer semantically consistent categories of sounds and images from the primary visual cortex through multivoxel pattern analysis. Another study successfully decoded four types of visual stimuli in retinal localization regions with the aid of sound modulation. These studies have shown that the information encoding of auditory information in the visual cortex is modulated by auditory information. Therefore, by combining the physical characteristics of different appearance elements and the target requirements of product appearance design, this paper proposes four quantitative mathematical models for product two-dimensional modeling, product three-dimensional modeling, product color, and product appearance integrating three-dimensional modeling and color.

This paper uses the RFX-BMS analysis method to find the model with the largest posterior probability from the 16 candidate models as the optimal model of the network. Model 12 has the highest excess probability (exceedance probability) of 0.61 among all models and is defined as the optimal model by us. The next best model is model 16, which has an excess probability of 0.19. The sum of the excess probabilities of the two is higher than 0.75, and the estimated optimal model is considered to be valid according to the rules of BMS. In model 12, STS, BA18, and HG all have bidirectional connections. This result suggests that the sensory cortex is subject to both top-down modulation from the higher processing area and reciprocal modulation between the sensory cortex.

### 3.2. Prediction of Modeling Image by Neural Network

*E*_1_, *E*_2_,…, *E*_*m*_ are the items in each representative sample. There are *n* car samples. The first item *E*_1_ has *r*_1_ categories, respectively: *E*_11_, *E*_12_,…, E_1*r*1_; the second item *E*_2_ has *r*_2_ categories: *E*_21_, *E*_22_,…, E_2*r*2_; then, the *m*th item *E*_*m*_ has *rm* categories, namely, *E*_*m*1_, *E*_*m*2_,…, *E*_*mrm*_. There are *p* categories in total. Among the samples, the response of the *k* category of the *j*th item is shown in the formula.

(1) $$\begin{array}{c} \delta_{i}\left(j,k\right)=\left\{\begin{array}{cc} 1, & i\in k,\\ 0, & i\notin k. \end{array}\right. \end{array}$$

Comparing 8 representative samples, “0” indicates that the design element does not include this category and “1” indicates that the design element includes this category. Therefore, the input data of the BP neural network are shown in Figure 2.

Representative car samples and 6 groups of adjectives were selected as representative samples for analysis.

1. Subject selection: 15 industrial design students with design background and 30 users without design background were selected to evaluate the samples.
2. Making a questionnaire survey: a perceptual image vocabulary evaluation table was made according to representative samples. The questionnaire survey used the semantic difference method (the scale was 7 steps), and the scale was scored from 1 to 7 from left to right.
3. Statistical analysis of data: the average value is obtained by analyzing and calculating according to the scale data.

DCM is to model the time evolution of the neural state vector of the brain region, and the changes in the brain neural state are mainly controlled by two external factors: the direct influence of the role and the specific region (direct influences) and the coupling of the mutual influence between regions. The strength of coupling among regions. The former is usually caused by direct experimental factors, such as the application of visual stimulation materials to the subjects in the experiment to evoke a response in the sensory cortex. The latter is usually elicited by high-level experimental tasks such as learning and attention tasks in experiments eliciting interregional reciprocity. In general, DMC models are estimates of neural states in the time domain. For *k* coupled brain regions, where *Z*_*k*_ represents the neural state in each brain region and *u* represents the external experimental input, the neural state equation in the entire region can be expressed as

(2) $$\begin{array}{c} |\begin{array}{c} Z1\\ Z2\\ Z3\\ ...\\ Zk \end{array}\rangle =\frac{\partial z}{\partial t}+\sum_{i=1}^{m}u_{i}B_{i}z+Cu. \end{array}$$

Among them, *A*, *B*, and *C* are the three basic causal components of neural state modeling: (1) *A* represents the endogenous connection parameters. They reflect the degree of context-independent coupling between neural states in different brain regions, such as mediated by anatomical connections between regions. (2) *B* represents the regulatory parameters. These parameters reflect the degree of influence on the effective connectivity of brain regions under the influence of external experimental input *u* (context-dependent), such as the degree of influence on brain regions under different experimental conditions. (3) *C* represents the driving input parameters. They reflect the degree to which brain regions respond directly to external experimental input *u*, such as the direct response of the sensory cortex to external stimuli. The neural dynamics model of DCM is shown in Figure 3, and the state equations of the three causal components are as follows. The STS has been mentioned several times in this paper as a key area of integration for the gathering of auditory and visual information. In the advanced frontoparietal control region, we selected three network nodes, namely, MFG, PFC, and IPL. From the activation results, both modalities have significant activation areas in the frontoparietal region, which also provides conditions for us to select network nodes.

(3) $$\begin{array}{c} A=\frac{\partial F}{\partial Z},\\ B_{j}=\frac{\partial^{2}F}{\partial Z\partial u_{j}}=\frac{\partial }{\partial u_{j}}\frac{\partial Z}{\partial u},\\ C=\frac{\partial Z}{\partial u}. \end{array}$$

In the process of DCM parameter estimation, Bayesian estimation is usually used to estimate the parameters of the candidate model. According to the Bayesian formula,

(4) $$\begin{array}{c} P\left(\theta |y\right)=P\left(y|\theta \right)P\left(\theta \right), \end{array}$$

where *P* is the prior knowledge of the parameter based on the experimental design, usually predefined by the researcher based on experience. It is the likelihood function of the prior distribution of the parameter. *Y* is the posterior distribution given the parameter. When estimating the parameters of the brain nodes, the posterior distribution of the assumed parameters is usually a Gaussian distribution, and the expectation-maximization algorithm is used at this time to estimate the parameter. We define the brain state equation as

(5) $$\begin{array}{c} x=f\left(x,u,\theta \right),\\ y=\lambda \left(x\right). \end{array}$$

Given the input signal *u* and the parameter *x*, the predicted value of the output signal can be obtained by integrating the equation.

We define this equation as the observation equation of the output signal, where *X* represents the task-independent amount of confusion, which is the observation error.

(6) $$\begin{array}{c} y=h\left(u,\theta \right)+\beta X+\omega . \end{array}$$

A local linear approximation can be obtained as follows:

(7) $$\begin{array}{c} y-h\left(u,\theta \right)=\beta X+\omega \approx J\Delta \theta +X+\varepsilon ,\\ \Delta \theta =\theta -J^{i},\\ J^{i}=\frac{\partial h\left(u,\theta \right)}{\partial \theta }. \end{array}$$

The posterior distribution of the parameter is assumed to be a Gaussian distribution by Bayes theorem, and the posterior distribution of the state *y* can be obtained as follows:

(8) $$\begin{array}{c} p\left(\theta \right)\in {\left(e^{-0.5\theta -\eta_{\theta |y}}\right)}^{T}e^{-0.5\theta -\eta_{\theta |y}},\\ C_{\theta |y}={\left(J^{T}C^{-1}J+C\right)}^{-1}. \end{array}$$

In the study of brain cognition, researchers usually find the activation region of interest through univariate analysis according to the experimental design, that is, select the ROI. Each ROI represents a node in the DCM network analysis. At this point, the researcher needs to predefine which nodes have possible connections and if so, what is the direction of the connection. In general, if there is relatively certain prior knowledge between the two nodes (for example, there is a proven anatomical connection between the nodes), the connection relationship between the two nodes can be determined; if the connection relationship between the nodes cannot be determined, it is necessary to traverse all possible connections, and all the permutations and combinations of these connections form the network space of the model, which is usually called a fully connected model space.

### 3.3. Determination of the Relationship between Modeling Image and User Satisfaction

The product modeling image is the user's emotional response triggered by the modeling part of the product appearance. Its positioning purpose is to determine the typical representative emotional response formed by the user to the overall modeling sample of the target product and to evaluate the data with several modeling target image adjectives and their perceptual images. The matrix is the quantized output of the positioning result. The scientific positioning of the modeling image is of great significance to the product image modeling design for user sensibility. The output data can truthfully reflect the diverse emotional needs of consumers for product modeling and provide reliable data-driven product appearance image design. Styling image data and clear design goals. The traditional product modeling image positioning process generally includes the following steps: (1) after determining the target product modeling sample, collect the perceptual vocabulary used to describe the sample modeling based on the survey data and interviews; (2) use the expert interview method and other technical means to carry out the perceptual vocabulary and conduct preliminary screening to reduce the number of words; (3) use the Likert scale method to evaluate the similarity of perceptual words and summarize the evaluation data to form a similarity matrix of perceptual words; (4) carry out cluster analysis on the similarity matrix of perceptual words and complete the modeling image positioning.

This positioning method relies too much on the subjective experience evaluation of the subjects, ignoring the use of the target product modeling data in the modeling image positioning process, and in the process and results of the cluster analysis, perceptual image information is lost and the multitarget image cannot be guaranteed. Coverage and failure reflect differences in importance between different target imagery. In order to better achieve the goal of modeling image positioning, this section incorporates the mathematical models of 2D modeling and 3D modeling quantification into the modeling image positioning process, uses the objective data obtained after modeling to participate in the construction of a modeling image comprehensive evaluation model, and finally realizes modeling imagery position. The positioning method includes determination of modeling sample set and modeling image vocabulary set, modeling quantitative mathematical description, modeling image measurement, modeling image comprehensive evaluation model construction, and modeling image positioning. The specific positioning process is shown in Figure 4.

The determination of the modeling sample set and the image vocabulary set is the first step in the positioning of the product modeling image, and it is also a very important link. Among them, the modeling sample set is a set composed of the modeling of several target products, and its determination often needs to consider the following factors: (1) the market segment of the target product. There are obvious differences in the product shapes and their perceptual expressions in different market segments. The research on the modeling image positioning of products belonging to the same market segment can better determine the goal and direction of product design and development. (2) The selected product sample shape should be typical. The overall modeling sample should reflect the whole picture of the target product market segment as much as possible, and the individual modeling samples should have obvious different modeling characteristics. (3) The final target product modeling sample determined should have good modeling quality and be able to clearly convey its own styling characteristics. In the actual determination process of the modeling sample set, we generally first try to select product samples that have a high market share in the target market segment and are familiar to consumers. The final samples are subjected to modeling preprocessing to form the final modeling sample set.

## 4. Design Perceptual Evaluation

The STS area is also a key area of this study, and the results of the previous chapters have found that the STS exhibits subsuperimposed integrated information in multisensory modulation and is a key location for the sensory cortex to receive top-down feedback. The results of functional connectivity allow us to further confirm the above results; the STS area is like a network hub, it receives information from the sensory cortex and projects to higher processing areas, which process the information and then funnel the information to the STS, which is finally fed back to the STS. Brain networks are selected at different processing levels and combined with prior knowledge, and four networks of animate and inanimate networks in the AVd mode and the Vd mode are, respectively, constructed. From the correlation coefficient matrix between network nodes, the positive correlation coefficients of the integration area in the AVd mode under the animate and inanimate categories are slightly higher than that in the Vd mode and are concentrated in the advanced frontoparietal control area, as shown in Figure 5. This suggests that auditory stimuli elicit more information transfer and integration between higher-order cortices in noisy image recognition, resulting in more frequent connections between these cortices. In order to see the changes in the network in different situations more clearly, we construct a positive and negative correlation network seed node connection graph. In the positive connection graph, anatomically close regions tend to have positive connections, such as BA18 and LOC, STS, and HG. The two nodes in the sensory cortex, BA18 and HG, have little or no connection to other areas except for the presence of connections to the STS. This indicates that the sensory cortex transmits and processes information according to levels and other integrated areas in the multimodal processing process; that is to say, the signals projected by the sensory cortex are generally transmitted step by step in the order of processing from primary to advanced, rather than directly with advanced cortical interactions. The positive correlation network characteristics conform to the “distributed-plus-hub” model proposed by recent scholars. There are fewer connections between nodes in the negative correlation network, and most of the connections appear in two areas that are basically unrelated to cognitive function, such as the sensory cortex BA18 and the MFG area of language and word processing.

Processing models at this level have been demonstrated. In addition, we also observed that PFC, STS, and LOC are nodes with a large number of positive connection relationships, especially the STS area, which is almost connected to most nodes, as shown in Figure 6. This processing mode has been confirmed by more and more studies in recent years. While the two regions, nodal PFC and LOC, are high-level regions for multimodal class processing, which is consistent with our experimental task. In fact, positively and negatively correlated functional connectivity is a reflection of the transmission of excitatory and inhibitory activity between neurons within the brain. Furthermore, comparing the positively correlated connection graphs of the animate and inanimate categories, the former has more connections in nodes at lower levels, for example, the link between BA18 and HG. This may be because animate categories are more familiar to us and the brain can recognize noise-added objects through lower-level processing, while inanimate categories are more difficult to identify, and lower-level processing areas cannot achieve recognition. Processing areas are consolidated.

In order to investigate the modulation mechanism of multimodality more comprehensively, we first selected multimodal integration regions as network nodes according to different processing levels before brain network analysis. Therefore, in the univariate analysis, this study firstly screened the network nodes one by one according to the activation results of the AVd mode and the Vd mode under the animate and inanimate categories and combined with the AAL template. Due to the limitations of the fMRI acquisition equipment, we did not consider the area of subcutaneous tissue. First, the BA18 and HG regions serve as visual and auditory unimodal cortical nodes, respectively. The LOC and STS regions are subadvanced joint processing regions, and the LOC region is widely regarded as the key region for visual object category processing. However, recent studies have shown that in the process of multisensory integration, LOC not only processes visual category information but also integrates information from other modalities such as touch and hearing, which is considered as a multimodal object category and shape perception area.

The frontoparietal region is the area of high-level cognitive processing. In our experiment, noise was added to the visual object and the subjects recognized the object with the assistance of semantically consistent sounds. Therefore, this process includes high-level cognition such as working memory and task decision-making process. The main purpose of applying these new methods to functional image data analysis is to reduce the dimension of features. In our study, another dimension of brain signal data was used as a feature (functional connectivity coefficient), and it was found that functional connectivity as a feature could significantly distinguish animate and inanimate categories, although the classification effect was not based on BOLD signal features. However, functional connections have the characteristics of small data dimensionality and low interference noise. Previous studies have confirmed the effectiveness of this method, but most of these studies extracted features by way of whole-brain functional connections, while this study predefines the nodes of the network based on prior knowledge, that is, reduces the number of network connection edges, and can also rule out the influence of some unrelated brain regions on category processing, as shown in Figure 7.

Harmonic techniques including elliptic Fourier and spherical harmonics demonstrate significant advantages in quantitative mathematical description of product shapes. Compared with other modeling quantification techniques, it improves the accuracy and freedom of modeling representation, as well as the accuracy and comprehensiveness of modeling image positioning. For the quantification of 3D modeling of products with complex surfaces, the amount of grid data and the difficulty in analysis and processing of 3D modeling are relatively large, but harmonic technology still has a good quantification capability for this object, as shown in Figure 8. By utilizing spherical parameters, spherical harmonics are very suitable for comprehensive quantitative processing and analysis of product 3D modeling. It can flexibly select high-frequency or low-frequency harmonics according to actual engineering needs to quantify the three-dimensional modeling of products and achieve a balance between fine effects and computational efficiency. By converting the grid data into uniform spherical harmonic coefficients, not only the normative data that are more concise and easier to achieve dimensionality reduction are obtained but also because the data volume of spherical harmonic coefficients is much smaller than that of grid data, the conversion process data dimensionality reduction has been achieved to a certain extent.

Product appearance includes three-dimensional modeling elements and color elements. Therefore, the product appearance image is formed by the characteristics of these two aspects of appearance elements, and the appearance element feature information is comprehensively represented by appearance data including multiple modeling principal component data and multiple color variable data. Due to the large number of variables in the appearance data, there is a more complex data mapping relationship between the multitarget image prediction of product appearance and the image value of each appearance target, in view of the predictive ability of multiple regression analysis technology to face such problems. Therefore, it is necessary to seek more applicable prediction techniques to establish an appearance image prediction model with good prediction effect. As shown in Figure 9, considering that the appearance variable data and the average appearance target image score as input and output variables are continuous data, the prediction and fitting ability of the back-propagation neural network to continuous data is better than that of multiple regression. The analysis technique is stronger and more stable, and the BPNN optimized by the genetic algorithm can better predict the nonlinear mapping relationship between input and output variables. Therefore, GABP is used as a prediction technique for the product appearance image prediction model.

## 5. Conclusion

The correction operator uses this relationship to adjust the evolution direction, thereby reducing the amount of computation and improving the efficiency and performance of ISPEA2 approximating the true Pareto scheme. When visual objects are disturbed in complex scenes, the issues such as how the human brain coordinates multisensory information processing and what neural processing mechanisms follow are still unclear. In this paper, a visual object recognition experiment in a complex scene was designed and the brain activation signals of three modalities of noise, added audio-visual (AVd), single visual noise and noise (Vd), and single-audio (A), were recorded by fMRI. The properties and neural processing mechanisms of multisensory modulation of auditory stimuli during noisy image recognition were explored. Using the conjunction method combined with the classic “max criterion” rule, it was found that only when a certain amount of noise was added to the visual stimulus, the integration area changed. Among them, the visual association area (BA18) showed super-superposition integration and the superior temporal sulcus (STS) area showed subsuperposition integration, confirming that both BA18 and STS regions were involved in the integration of multimodal information under visual noise addition. In addition, pattern analysis of brain activation signals confirmed that semantically consistent sounds can facilitate the recognition of noisy images, and this facilitation shows a certain category selectivity when subdivided into categories. Using the analysis method of functional connectivity, a functional connectivity network containing nodes at different integration levels was constructed to explore the overall characteristics and processing patterns of the multisensory network. Through the analysis of the network connection relationship, it is found that the prefrontal cortex, STS, and lateral occipital lobe are the nodes with more aggregation in the network, and their functions are like the hub in the network. In addition, BA18 and HG have little connection to other regions except that they are connected to each other and to STS.

## Figures and Tables

**Figure 1:** Multimodal modeling design of product modeling.

**Figure 2:** BP neural network input data.

**Figure 3:** Multiple value additions and enhancements.

**Figure 4:** Product image positioning. (a) Image. (b) Modeling image.

**Figure 5:** Classification results of different feature selection methods.

**Figure 6:** Comparison of classification accuracy under two feature selections.

**Figure 7:** Brain regions significantly activated by the three ROIs.

**Figure 8:** Comprehensive quantification of product 3D modeling. (a) Appearance. (b) Target. (c) Prediction.

**Figure 9:** Appearance intention prediction model.

## Data Availability

The data used to support the findings of this study are available from the corresponding author upon request.
